# Chitosan-Coated Titanium Dioxide-Embedded Paclitaxel Nanoparticles Enhance Anti-Tumor Efficacy Against Osteosarcoma

This article has been retracted.

**DOI:** 10.3389/fonc.2020.577280

**Published:** 2020-09-09

**Authors:** Yang Qu, Mingyang Kang, Xueliang Cheng, Jianwu Zhao

**Affiliations:** Department of Orthopedics, The Second Hospital of Jilin University, Changchun, China

**Keywords:** osteosarcoma, titanium dioxide nanoparticles, chitosan, antioxidant, anti-inflammatory, anti-tumor, survival rate

## Abstract

**Objective:**

Titanium dioxide nanoparticles (TiO_2_) nanoparticles have been widely explored in the prevention of cancer risk. Due to the difficult solubility of TiO_2_ nanoparticles, it is essential to synthesize new surfactants to increase its bioavailability and anti-tumor activity and reduce its cytotoxicity. Furthermore, oxidative and inflammation are closely associated with the osteosarcoma risk. Chitosan has biocompatibility, antioxidant and anti-inflammatory properties. The effects of chitosan-coated TiO_2_-embedded paclitaxel nanoparticles on an osteosarcoma model were explored.

**Methods:**

An osteosarcoma model was established and chitosan-coated TiO_2_-embedded paclitaxel nanoparticles were prepared using a freeze-drying strategy. The morphological characteristics of nanoparticles were observed using scanning electron microscopy (SEM). The physicochemical properties of nanoparticle were evaluated by X-ray diffraction (XRD) and Fourier transform infrared (FTIR) spectroscopy. The cytotoxicity was tested by using human osteoblast cells hFob1.19 and osteosarcoma cells 143B. Osteosarcoma mice were treated with PBS buffer, paclitaxel, TiO_2_-embedded paclitaxel and chitosan-coated TiO_2_-embedded paclitaxel nanoparticles. The biomarkers of oxidative-inflammatory status, anti-tumor activities and survival rates of the model were measured.

**Results:**

XRD analysis showed that the peaks of chitosan/TiO_2_ (anatase) were consistent with those of crystalline TiO_2_ and broad phase of chitosan. The FTIR spectrum indicated the relevant functional groups in TiO_2_. Chitosan-coated TiO_2_-embedded paclitaxel nanoparticles had good biocompatibility and improve antioxidant and anti-inflammatory properties in the osteosarcoma model. Chitosan-coated TiO_2_-embedded paclitaxel nanoparticles was less toxic to the cells hFob1.19 and more toxic to the cells 143B than TiO_2_-embedded paclitaxel nanoparticles. Chitosan-coated TiO_2_-embedded paclitaxel nanoparticles showed significant antitumor activity and increased the survival rate of the osteosarcoma model (*P* < 0.05).

**Conclusions:**

Chitosan improved anti-tumor potential of TiO_2_-embedded paclitaxel nanoparticles in the prevention of osteosarcoma.

## Introduction

Osteosarcoma is the leading cause of bone malignancy (1) and one of the important causes of death and disability worldwide (2, 3). The disease is a common emergency in bone surgery and should be early diagnosed and treated to obtain a better prognosis. Titanium dioxide (TiO_2_) nanoparticles are potential materials in the prevention of osteosarcoma and chondrosarcoma recurrence (4). Paclitaxel, classified as a “plant alkaloid,” is isolated originally from the bark of *Taxus brevifolia* and has been widely reported in the treatment of osteosarcoma (5, 6). TiO_2_-embedded paclitaxel nanoparticles have been tried in the prevention of cancer risk (7). However, due to the difficult solubility of paclitaxel, it is essential to explore new forms to increase its bioavailability and anti-tumor activity and reduce toxicity (8, 9).

Chitosan, a promising natural polysaccharide and the derivative of chitin, is used as a friendly biomaterial in tissue engineering because of its biocompatibility and easy degradation without toxicity (10, 11). Chitosan polymeric micelles have been developed for improving the bioavailability of paclitaxel and reducing its toxicity (12–14). However, chitosan has various disadvantages, such as weak mechanical strength (15, 16) and fast degradation (17). TiO_2_ is available in nanocrystals with wide surface area and has antibacterial activity (18). TiO_2_ has been used as good material in medical and health applications due to its inert property (19). Chitosan molecules can be assembled through hydrophobic interaction and hydrogen binding (20). Both chitosan and TiO_2_ are biocompatible, inert, and chemically stable so that they may be beneficial in the prevention of osteosarcoma progression.

Oxidative stress often induces osteosarcoma cell invasion, migration, and the epithelial-to-mesenchymal transition through the miR-153/snail family zinc finger 1 axis (21). Furthermore, pretreatment inflammatory index neutrophil-lymphocyte ratio is associated with the poor outcomes in patients (22). Thus, the antioxidant and anti-inflammatory therapy is a potential approach in the prevention of the progression and development of osteosarcoma (23, 24). Fortunately, the antioxidant and anti-inflammatory properties of chitosan have been widely reported (25, 26).

The purpose of this study is to compare the properties of chitosan-coated TiO_2_-embedded paclitaxel nanoparticles and TiO_2_-embedded paclitaxel nanoparticles and analyze the effects of chitosan in the prevention of osteosarcoma development.

## Materials and Methods

### Synthesis of Chitosan-Coated TiO_2_-Embedded Paclitaxel and TiO_2_-Embedded Paclitaxel Nanoparticles

Low-molecular-weight chitosan (80% deacetylated) was purchased from Aokang Biotech Co., China. TiO_2_-embedded paclitaxel nanoparticles were purchased from Grikin (Beijing, China). TiO_2_-embedded paclitaxel nanoparticles were synthesized by using grafting folic acid for targeted paclitaxel onto TiO_2_ as nanocarrier. Different concentrations of chitosan acetic acid hydrosol was prepared by the dissolution of 20, 40, 60, and 80 g chitosan powder into 200-ml ddH_2_O with 2-ml acetic acid. Chitosan in an acidic solution was sprayed and dispersed via a spray drying technology, and then sprayed in a hot gas stream to rapidly form chitosan-coated TiO_2_-embedded paclitaxel nanoparticles.

### SEM Observation

Scanning electron microscopy (SEM) is a common technique to characterize the morphology, and size of nanoparticles (27–31), and was conducted on JEOL JSM 5900LV [JEOL (Beijing) Co., Ltd., Beijing, China]. SEM showed morphological characteristics of TiO_2_-embedded paclitaxel and chitosan-coated TiO_2_-embedded paclitaxel nanoparticles. For the SEM analysis, the nanoparticles were covered with gold coating and observed via the Scanning Electroscope JEOL JSM 5900LV. Meanwhile, the microstructure of two kinds of nanoparticles was examined with SEM. The Energy Dispersive X-Ray Spectroscopy (EDS) spectra were developed using JEOL SEM (20 kV).

### XRD Analysis

X-ray diffraction (XRD) has become a routine method to measure the structure and phase and crystallinity and purity of nanoparticles (27–32). The structure and phase TiO_2_ and chitosan-coated TiO_2_ nanoparticles were characterized by XRD. The diffraction pattern of TiO_2_ sample was indexed by comparing with the anatase TiO_2_ and rutile TiO_2_ standards from Sigma-Aldrich and the Joint Committee on Powder Diffraction Standards (JCPDS) Card File No. 21-1272 and 21-1276 (33). The graphical X-ray powder diffraction patterns of the TiO_2_-embedded paclitaxel and chitosan-coated TiO_2_-embedded paclitaxel samples were observed by using Ultima IV X-ray diffractometer (Rigaku, Woodlands, TX, United States), using Cu-Ka (1.5 Å) in the range of 20° to 60° at 2θ degree. XRD analysis was adjusted according to the anatase TiO_2_ and rutile TiO_2_ standards.

### FTIR Analysis

FTIR spectra (from 4,000 to 500 cm^–1^) of the surface of TiO_2_-embedded paclitaxel and chitosan-coated TiO_2_-embedded paclitaxel nanoparticles were measured in Perkin Elmer Spectrum RX1 spectrometer (Canton, MA, United States). FTIR showed the related functional groups in the molecules.

### MTT [3-(4,5-Dimethylthiazol-2-yl)-2, 5-Diphenyltetrazolium Bromide] Analysis of the Toxicity of Chitosan-Coated TiO_2_-Embedded Paclitaxel and TiO_2_-Embedded Paclitaxel Nanoparticles

The human osteoblast cells hFob1.19 and osteosarcoma cells 143B were purchased from the cell bank of Shanghai Institutes for Biological Sciences (Shanghai, China) and cultured in DMEM medium (Gibco, Shanghai, China) supplemented with 10% heat-inactivated FBS (Hyclone, Shanghai, China), 100 μg/mL of penicillin and 100 μg/mL of streptomycin (Yuanmu Biotechnology Co., Ltd., Shanghai, China). All cells were cultured at 37°C in a 5% CO_2_ atmosphere. The culture temperature of hFob1.19 cell was 33.5°C, and 143B cell was 37°C. The cells were transferred into a 96-well plate at a cell density of 1 × 10^4^ cells/well with 5% CO_2_. After culturing for 24 h, 50 μL of different concentrations of paclitaxel, chitosan-coated TiO_2_-embedded paclitaxel or TiO_2_-embedded paclitaxel nanoparticles were added after the cells fully adhered. The final concentration gradients of paclitaxel were 0.36, 0.725, 0.15, 0.31, 0.625, 1.25, 2.5, 5, and 10 μg/mL. The 96-well plate was placed in the cell incubator and continued to be incubated for 72 h, and then 20 μL of pre-configured MTT (Sigma-Aldrich, St. Louis, MO, United States) PBS solution was added to each well and continued to be incubated for 4 h. Subsequently, the medium in each well was carefully removed and 200 μL of DMSO was added and shaken for 10 min to completely dissolve the blue-violet formazan. Finally, the absorbance value (A) at 490 nm was measured with a microplate reader to calculate the cell survival rate. Cell viability was calculated as follows: (OD values in experimental wells-OD values in blank wells)/(OD values in control wells - OD values in blank wells) × 100.

### Animal Grouping and Establishment of Osteosarcoma Model

Before the experiments, all procedures were approved by the animal research ethics committee of The Second Hospital of Jilin University (Approval No. 2019JLU23D). Forty-eight female BALB-c nude mice (4 weeks, 18–22 g) were purchased from the animal center of Jilin University (Changchun, China) and randomly divided into four groups on average: control group (PBS solution, CG), experimental group chitosan-coated TiO_2_-embedded paclitaxel (5 mg/kg) nanoparticles (PCTG), paclitaxel (PG, 5 mg/kg), TiO_2_-embedded paclitaxel (5 mg/kg) nanoparticles (PTG), first adapt to the environment and trained for 2 weeks. Nude mice were anesthetized by intraperitoneal ketamine/xylazine (100 mg per kg/10 mg per kg) (34). After the nude mice enter anesthesia, follow-up operations are performed. After anesthetizing nude mice, 50 μL 1 × 10^7^ cells/mL 143B-luc suspension was injected into the proximal tibia of each nude mouse with a 25-G needle. After the tumor cells were inoculated, each nude mouse was randomly checked for tumor formation in the tibia of the left lower limb. Osteosarcoma is relatively deep, so it is impossible to determine whether a tumor has formed by visual inspection and touch. 143B cells can generally form tumors *in situ* in 2 weeks, and the positive fluorescence signal in live imaging is the standard for tumor formation.

### Measurement of Markers of Oxidative-Inflammatory Status

A sample of 0.5 ml of blood was obtained from the mouse tail vein. The serum was prepared via centrifugation at 2,000 × *g* for 10 min and stored at −20°C for ELISA measurement. Serum tumor necrosis factor α (TNFα) (ab208348), interleukin (IL)-1 β (ab100705), IL-6 (ab222503) and IL-10 (ab255729) were examined using the ELISA kits from Abcam (Cambridge, MA, United States). Serum superoxide dismutase (SOD) (MBS034842) and catalase (CAT) (MBS704962), glutathione peroxidase (GSPx) (MBS723759) and MDA (MBS741034) were determined using the kits from MyBioSource, Inc. (Vancouver, WA, United States). All these biomarkers were measured on an automatic chemical analyzer (CliniTek 500, Bayer, United States).

### *In vivo* Imaging of Osteosarcoma

After 14-day tumor cell inoculation, different groups of nude mice were treated with PBS buffer, paclitaxel, chitosan-coated TiO_2_-embedded paclitaxel nanoparticles or TiO_2_-embedded paclitaxel nanoparticles, respectively. The dose of paclitaxel was 5 mg/kg in the 3 latter groups (35). Subsequently, nude mice received *in situ* tumor injection treatment twice a week. On days 14, 21, and 28, live imaging was performed on nude mice and fluorescein was injected before 5-min imaging. The nude mice were anesthetized after 15–20 min of activity, and placed in the prone position in the imaging detection system. In the statistical analysis, the tumor bioluminescence intensity was normalized to the initial amount of fluorescence intensity on the 14th day of each nude mouse.

### Tumor Mass

After 28 days of tumor cell inoculation, the nude mice of each group were imaged *in vivo*. The nude mice were sacrificed, osteosarcoma tissue was dissected, washed with PBS, and cleaned with filter paper. The tumor mass was evaluated among different groups.

### Survival Curve of the Mice

To investigate the survival curves of the nude mice of the control group (PBS solution) and the experimental groups, *in situ* injection therapy was performed twice a week after 2 weeks of injection of 143B cells. During the treatment, the survival rate was calculated every week for 10 weeks among another four groups: control group (PBS solution, CG), experimental group chitosan-coated TiO_2_-embedded paclitaxel (5 mg/kg) nanoparticles (PCTG), paclitaxel (PG, 5 mg/kg), and TiO_2_-embedded paclitaxel (5 mg/kg) nanoparticles (PTG).

### Statistical Analysis

The data were presented as mean values ± standard deviation (SD). The normal distribution was analyzed using the Shapiro-Wilk test and a two-tailed Student’s *t*-test was used to compare the significance of two groups. The count data were analyzed by a chi-square test. *P* < 0.05 was considered statistically significant.

## Results

### Morphologic Characters of Chitosan Nanoparticles

The maps of all samples were shown in Supplementary Figure S1. SEM showed that TiO_2_-embedded paclitaxel nanoparticles were spherical and the diameter of TiO_2_-embedded paclitaxel nanoparticles ranged from 40 to 60 nm (Figures 1a,b). EDS was used to characterize the elemental composition of chitosan-coated TiO_2_ nanoparticles prepared by using different concentration of chitosan. In the TiO_2_ nanoparticles, the main elements O and Ti were observed (Figure 1c), which were consistent with the main elements of TiO_2_ nanoparticle. SEM of chitosan-coated TiO_2_-embedded paclitaxel nanoparticles with the size from 40 to 200 nm presented a spherical shape with some irregular shapes. With the increase in the concentration of chitosan, the size of nanoparticles increased. The diameter ranged from 40 to 80 nm for 1% chitosan-coated TiO_2_-embedded paclitaxel nanoparticles (Figures 1d,e), from 40 to 120 nm for 2% chitosan-coated TiO_2_-embedded paclitaxel nanoparticles (Figures 1g,h), from 40 to 160 nm for 3% chitosan-coated TiO_2_-embedded paclitaxel nanoparticles (Figures 1j,k), and from 40 to 200 nm for 4% chitosan-coated TiO_2_-embedded paclitaxel nanoparticles (Figures 1m,n). Large particles made a smooth area but the higher concentration of chitosan became difficult to be dissolved. Thus, 4% chitosan was used for the preparation of nanoparticles. The microstructure of nanoparticles was similar between non-coated and chitosan-coated ones. In the chitosan-coated TiO_2_ nanoparticles, the main elements C, N, O, Na, and Ti were observed (Figures 1f,i,l,o), which were consistent with the main elements of chitosan-coated TiO_2_ nanoparticle.

**FIGURE 1:** Scanning electron microscopy (SEM) analysis of TiO_2_-embedded paclitaxel nanoparticles and chitosan-coated TiO_2_ nanoparticles. **(a)** Micrograph of TiO_2_-embedded paclitaxel nanoparticles powder. **(b)** The size of TiO_2_-embedded paclitaxel nanoparticles powder. **(c)** Energy Dispersive X-Ray Spectroscopy (EDS) spectra for the TiO_2_ nanoparticle composite. **(d)** Micrograph of 1% chitosan-coated TiO_2_ oligosaccharides powder. **(e)** The size of 1% chitosan-coated TiO_2_-embedded paclitaxel nanoparticles powder. **(f)** EDS spectra for 1% chitosan-coated TiO_2_-embedded paclitaxel nanoparticles powder. **(g)** Micrograph of 2% chitosan-coated TiO_2_ oligosaccharides powder. **(h)** The size of 2% chitosan-coated TiO_2_-embedded paclitaxel nanoparticles powder. **(i)** EDS spectra for 2% chitosan-coated TiO_2_-embedded paclitaxel nanoparticles powder. **(j)** Micrograph of 3% chitosan-coated TiO_2_ oligosaccharides powder. **(k)** The size of 3% chitosan-coated TiO_2_-embedded paclitaxel nanoparticles powder. **(l)** EDS spectra for 3% chitosan-coated TiO_2_-embedded paclitaxel nanoparticles powder. **(m)** Micrograph of 4% chitosan-coated TiO_2_ oligosaccharides powder. **(n)** The size of 4% chitosan-coated TiO_2_-embedded paclitaxel nanoparticles powder. **(o)** EDS spectra for 4% chitosan-coated TiO_2_-embedded paclitaxel nanoparticles powder.

### Characterization of Chitosan-Coated TiO_2_-Embedded Paclitaxel Nanoparticles and TiO_2_ Nanoparticles

XRD analysis showed that the phase of TiO_2_ was the same as that of anatase TiO_2_ standard and JCPDS No. 21-1272. Thus, anatase TiO_2_ was used in the present nanoparticles. The peaks of chitosan-coated TiO_2_-embedded paclitaxel nanoparticles and TiO_2_-embedded paclitaxel nanoparticles at 25.1°, 36.9°, 37.9°, 38.8°, 48.0°, 54.0°, and 55.0° corresponding to TiO_2_ (crystalline) and broad phase 30.0°, 36.0°, 43.4°, 54.5° and 58.0° corresponding to chitosan (Figure 2A). The results suggest that chitosan has excellent physiochemical properties such as biocompatible.

**FIGURE 2:** Characterization of chitosan-coated TiO_2_-embedded paclitaxel nanoparticles and TiO_2_ nanoparticles. **(A)** XRD analysis of chitosan-coated TiO_2_ nanoparticles, chitosan and TiO_2_ nanoparticles. **(B)** FTIR analysis of chitosan-coated TiO_2_-embedded paclitaxel nanoparticles and TiO_2_ nanoparticles.

The FTIR spectrum indicated the relevant functional groups in chitosan-coated TiO_2_-embedded paclitaxel nanoparticles and TiO_2_-embedded paclitaxel nanoparticles (Figure 2B). There was a band present from 3,350 to 3,600 cm^–1^ because of OH vibrations. The band presented from 500 to 891 cm^–1^ for Ti–O–Ti vibrations, 1,630 cm^–1^ showed Ti-OH vibrations because of adsorbed H_2_O and 1,380 cm^–1^ indicated Ti-O. The functional groups C-H and C = O were detected at peaks 2,942 and 1,656 cm^–1^, respectively.

### MTT Cytotoxicity Evaluation

The cytotoxicity of nanoparticles and paclitaxel was evaluated by the MTT method. As shown in Figure 3A for the human osteoblast cell line hFob1.19, with the increase in the concentration of paclitaxel, TiO_2_-embedded paclitaxel and chitosan-coated TiO_2_ nanoparticles, the cytotoxicity was enhanced. When the drug concentration was more than 10 μg/mL, the cell survival rate was still more than 80%, which was between TiO_2_-embedded paclitaxel and chitosan-coated TiO_2_ nanoparticles. In the present study, the paclitaxel concentration 5 μg/mL (5 mg/kg) was selected to be used in the model. As shown in Figure 3B, for the human osteosarcoma cell line (143B), paclitaxel, TiO_2_-embedded paclitaxel and chitosan-coated TiO_2_-embedded paclitaxel nanoparticles all had growth-inhibiting effects on the cell growth, and chitosan-coated TiO_2_-embedded paclitaxel nanoparticles were the most toxic to the cells 143B in a concentration-dependent way. The experimental results show that chitosan-coated TiO_2_-embedded paclitaxel nanoparticles have good biocompatibility with normal human osteoblasts and a certain growth inhibitory effect on human osteosarcoma cell lines.

**FIGURE 3:** MTT assay was used to evaluate the toxicity *in vitro* of paclitaxel and or nanoparticle-embedded paclitaxel on **(A)** hFob1.19 cells and **(B)** 143B cells. There were four groups: control group (CG), paclitaxel group (PG), TiO_2_-embedded paclitaxel nanoparticle group (PTG), and chitosan-coated TiO_2_-embedded paclitaxel nanoparticles (PCTG). The cell viability was regarded 100% in the CG group. *n* = 8 for each group.

### Chitosan Increased Antioxidant and Anti-inflammatory Properties

After the establishment of the osteosarcoma model, the levels of SOD (Figure 4A), CAT (Figure 4B), and GSPx (Figure 4C) were decreased while MDA (Figure 4D) was increased in the CG group when compared with the other groups (*P* < 0.05). Paclitaxel, TiO_2_-embedded paclitaxel and chitosan-coated TiO_2_-embedded paclitaxel nanoparticles treatment increased the levels of SOD (Figure 4A), CAT (Figure 4B), and GSPx (Figure 4C) and reduced the level of MDA (Figure 4D, *P* < 0.05). Especially, chitosan-coated TiO_2_-embedded paclitaxel nanoparticles caused the changes of oxidative stress biomarkers higher than those in other groups (Figure 4, *P* < 0.05).

**FIGURE 4:** The effects of chitosan on the levels of oxidative stress biomarkers. **(A)** SOD. **(B)** CAT. **(C)** GSPx. **(D)** MDA. *n* = 8 for each group. ^a^*P* < 0.05 vs the CG group, ^b^*P* < 0.05 vs the PG group, ^c^*P* < 0.05 vs the PTG group and ^d^*P* < 0.05 vs the PCTG group.

After the establishment of osteosarcoma model, the levels of TNFα (Figure 5A), IL-1 (Figure 5B), and IL-6 (Figure 5C) increased while the level of IL-10 (Figure 5D) reduced in the CG group when compared with the other groups (*P* < 0.05). Paclitaxel, TiO_2_-embedded paclitaxel and chitosan-coated TiO_2_-embedded paclitaxel nanoparticles treatment reduced the level of TNFα (Figure 5A), IL-1 (Figure 5B), and IL-6 (Figure 5C) and increased the level of IL-10 (Figure 5D, *P* < 0.05). Especially, chitosan-coated TiO_2_-embedded paclitaxel nanoparticles caused the changes in inflammatory cytokines higher than that in the SG group (Figure 5D, *P* < 0.05). All these results suggest that chitosan increases antioxidant and anti-inflammatory properties.

**FIGURE 5:** The effects of chitosan decoction on the levels of inflammatory cytokines. **(A)** TNFα. **(B)** IL-1β. **(C)** IL-6. **(D)** IL-10. *n* = 8 for each group. ^a^*P* < 0.05 vs the CG group, ^b^*P* < 0.05 vs the PG group, ^c^*P* < 0.05 vs the PTG group and ^d^*P* < 0.05 vs the PCTG group.

### Evaluation of Antitumor Effect *in vivo*

After 14 days of the inoculation of 143B cells, the nude mice from different groups were subjected to bioluminescence imaging to confirm that *in situ* tumors had formed. As shown in Figure 6, each group had obvious fluorescence imaging near the inoculated cells, indicating that the *in situ* osteosarcoma model was established successfully; the fluorescence area of the tumor site gradually expanded with the nude mice grew in the CG group; after the treatment of chitosan-coated TiO_2_-embedded paclitaxel nanoparticles treatment in the PTCG, the fluorescent area of the tumor site gradually reduced, indicating that the nanoparticles had a significant therapeutic effect on osteosarcoma; other experimental groups paclitaxel and TiO_2_-embedded paclitaxel has a certain treatment on osteosarcoma, but their inhibitory effects on the tumor were lower than that in the PCTG. Further work is needed to confirm these results.

**FIGURE 6:** Bioluminescence images of mice from each treatment group: control group (CG), paclitaxel group (PG), TiO_2_-embedded paclitaxelnanoparticle group (PTG), and chitosan-coated TiO_2_-embedded paclitaxel nanoparticles (PCTG). The mice from the different treatment groups at 14, 21, and 28 days; The statistical results were analyzed after normalizing tumor bioluminescence in each mouse to the initial flux. *n* = 8 for each group. ^a^*P* < 0.05 vs the CG group, ^b^*P* < 0.05 vs the PG group, ^c^*P* < 0.05 vs the PTG group and ^d^*P* < 0.05 vs the PCTG group.

After 28 days of tumor cell inoculation, the nude mice were sacrificed and the osteosarcoma tissues were shown in Figure 7. The growth rate of osteosarcoma could be controlled well in the PTCG group (*P* < 0.05). Comparatively, the growth was less controlled in the PG and PTG groups when compared with the PTCG group (*P* < 0.05). Chitosan and TiO_2_ may have synergistic function in the prevention of osteosarcoma growth. Chitosan-coated TiO_2_-embedded paclitaxel nanoparticles had the slow drug-release ability, which maintained the efficacy of drugs for a longer time and improved the therapeutic results.

**FIGURE 7:** The gross observation photographs of osteosarcoma tissue in different groups after treatment: control group (CG), paclitaxel group (PG), TiO_2_-embedded paclitaxelnanoparticle group (PTG), and chitosan-coated TiO_2_-embedded paclitaxel nanoparticles (PCTG). The tumor from the different treatment groups at 28 days; The statistical results were analyzed after normalizing tumor mass in the CG group. *n* = 8 for each group. ^a^*P* < 0.05 vs the CG group, ^b^*P* < 0.05 vs the PG group, ^c^*P* < 0.05 vs the PTG group and ^d^*P* < 0.05 vs the PCTG group.

### Chitosan Increased the Survival Rate of Osteosarcoma Model

The survival time of the nude mice among different groups was shown in Figure 8. It was found that the survival time of nude mice after intra-tumor injection of chitosan-coated TiO_2_-embedded paclitaxel nanoparticles was greatly prolonged, while the nude mice in the CG group most died at the 10 weeks. The results suggest that chitosan increased the survival rate of osteosarcoma model.

**FIGURE 8:** The survival rate of nude mice among different groups. control group (CG), paclitaxel group (PG), TiO_2_-embedded paclitaxelnanoparticle group (PTG), and chitosan-coated TiO_2_-embedded paclitaxel nanoparticles (PCTG). The tumor from the different treatment groups at 28 days; The statistical results were analyzed after normalizing tumor mass in the CG group. *n* = 8 for each group.

## Discussion

The synthesis of chitosan-coated nanoparticles meets the concept of green chemistry. Green synthesis of nanoparticles is the present topic of material research (36). This article focused on the construction of paclitaxel self-assembled nanodrugs based on the formation of assemblies between paclitaxel molecules chitosan and TiO_2_ molecules through hydrophilic/hydrophobic interactions and hydrogen bonding, etc. The addition of chitosan co-precipitated formed an assembly of three molecules because of its biocompatibility. There are modifiable sites on the paclitaxel molecule, which can be amphiphilic with TiO_2_. To construct a delivery system of hydroxyapatite-chitosan and TiO_2_-embedded paclitaxel nanoparticles for the treatment of osteosarcoma, chitosan was added after the synthesis of TiO_2_-embedded paclitaxel nanoparticles. The chitosan-coated TiO_2_-embedded paclitaxel nanoparticles using the freeze-drying technique exerted low density with nice mechanical characteristics. The notable adsorption or water holding activity of chitosan-coated TiO_2_-embedded paclitaxel nanoparticle was observed in the present experiment. Chitosan-coated TiO_2_ could be utilized for creating a biocompatible implant with low density. Biocompatible property of chitosan supported cells attachment, proliferation, and mineralization. TiO_2_ is inert, so the combination of chitosan/TiO_2_ can be a good substitute for tissue engineering. Further work is highly demanded to optimize numerous parameters of the chitosan-coated TiO_2_-embedded paclitaxel nanoparticles without compromising biodegradability and intoxicity. Multidisciplinary approach is also expected to fabricate novel nanoparticles with improved properties. The nanoparticles participated effectively eliminated osteosarcoma cells near bone tissue and prevented its development. Chitosan-coated TiO_2_-embedded paclitaxel nanoparticles had high drug-loading efficiency, and paclitaxel release lasts more than 5 days in the *in vitro* drug sustained-release experiment (data were not shown).

The present findings demonstrate that diameter of TiO_2_-embedded paclitaxel nanoparticles increases with the increase in the concentration of chitosan and the increase in the nanoparticle size has a linear relationship with the increase in chitosan concentration (Figure 1, The diameter ranged from 40 nm to 80/120/160/200 nm for 1%/2%/3%/4% chitosan-coated TiO_2_-embedded paclitaxel nanoparticles, respectively. The result is consistent with the previous report that the size of chitosan nanoparticles is mostly affected by the chitosan solution concentration, and the increase in nanoparticle size has a linear relationship with the increase in chitosan concentration (37). The size and surface charge of nanoparticles are important properties to understand their implications for possible biological impacts (38). Chitosan nanoparticles have positive charged surfaces and controlled sized according to chitosan concentration, suggesting that chitosan is potential biomaterial for developing nanoparticle-based drug carriers.

*In vitro* cell experiments showed that chitosan-coated TiO_2_-embedded paclitaxel nanoparticles had good biocompatibility and were effective in the prevention of osteosarcoma cell proliferation. The *in vivo* anti-tumor effect of chitosan-coated TiO_2_-embedded paclitaxel nanoparticles was evaluated using a nude mouse model of osteosarcoma *in situ*. Its anti-tumor effect was significant and it prevented tumor metastasis (Figure 6). The paclitaxel self-assembled Nano-drug delivery system was successfully constructed, characterized and showed anti-tumor properties. After the establishment of the osteosarcoma model, the inflammatory and oxidative stress activities were increased (Figures 4, 5), suggesting that inflammatory and oxidative responses were associated with osteosarcoma risk. Chitosan-coated TiO_2_-embedded paclitaxel nanoparticles protected the mice against osteosarcoma development by increasing antioxidant and anti-inflammatory capacities. All these results indicate that chitosan addition improves the biocompatibility, antioxidant and anti-inflammatory properties of TiO_2_-embedded paclitaxel nanoparticles in the osteosarcoma model. Meanwhile, chitosan addition increases the antitumor activity of TiO_2_-embedded paclitaxel nanoparticles and the survival rate of the osteosarcoma model.

Nanoparticle therapy has caught enormous interests in the treatment of tumors with multidrug resistance because of its synergistic effects focusing on tumor target cells and reduction of side effects on normal cells (39). Chitosan has been widely used as healthy products in China. The dosage of chitosan less than 1 g/kg b.w. will not affect autonomic or behavioral responses in an animal model (40). The present test showed that 40 mg/mL chitosan didn’t affect the viability of osteoblast cells.

In recent years, the research on chitosan has been widely carried out in drug development and delivery (41–44). It has been documented that chitosan nanoparticles have functions such as better regulation of the immune system and inhibition of tumor growth (45, 46). It can not only regulate the microbial metabolism in the intestine, but also regulate the micro-ecological environment (47, 48). It can lower blood pressure (49, 50), blood lipids, cholesterol (51), and chitosan nanoparticles have anti-oxidation and anti-inflammatory effects (52–54). Chitosan nanoparticles inhibit the growth of tumor cells by inducing cell necrosis and apoptosis (55, 56). The nanoparticles also reduce tumor angiogenesis to inhibit tumor cell metastasis (57, 58), and may also enhance human immunity. Chitosan should be developed a potential drug-delivering material to prevent osteosarcoma development.

There were some limitations to the present work: this study did not examine the repair of bone defects caused by osteosarcoma after surgery. The self-assembled morphology of chitosan-coated TiO_2_-embedded paclitaxel nanoparticles was rather special and there was no in-depth study on the presence of paclitaxel in the nanoparticles. The synergistic effect of chitosan and TiO_2_ and the mechanism of toxicity to osteosarcoma cells were not explored. The methods of chitosan-coated TiO_2_-embedded paclitaxel in this paper can be further optimized, which can further improve the drug loading. Thermosensitive hydrogels are hoped to be ideal materials for long-term controlling drug release. The mixture of hydrophilic polymer poly (vinyl alcohol) (PVA) and thermosensitive hydrogel composed of chitosan and glycerophosphate, can reduce body responses and increase the drug bioavailability (59). The hydrogelation of chitosan displays the phase transition from solution to hydrogel at body temperature (37°C) and body pH with β-GP (60). The temperature responsiveness of the chitosan-coated nanoparticle will promote drug release (61). High-Resolution Transmission Electron Microscopy (HRTEM) has become a routine tool in nanoparticle imaging and structure analysis. Atomic force microscopy can be used to analyze non-ideal conditions of these nanoparticles. Thermal characterization of nanomaterials was not undertaken, such as thermogravimetric analysis-differential thermal analysis (TGA-DTA), differential scanning calorimetry (DSC) and Derivative Thermogravimetric Analysis (DTG). These parameters are very important to acquire knowledge of the behavior of these nanoparticles under certain physiological temperature. Unfortunately, all the related work was not explored in the present paper. The current preparation conditions were based on the laboratory level, and further work was still needed to address these important issues.

## Conclusion

Chitosan was an important polymer with a wide range of applications in the therapy of osteosarcoma. The microstructure of chitosan-coated TiO_2_-embedded paclitaxel nanoparticles and TiO_2_ were consistent with the crystalline of TiO_2_ and broad phase of chitosan with relevant functional groups in TiO_2_ nanoparticles. Chitosan-coated TiO_2_-embedded paclitaxel nanoparticles increased antioxidant and anti-inflammatory, and anti-tumor properties.

## Data Availability Statement

The raw data supporting the conclusions of this article will be made available by the authors, without undue reservation.

## Ethics Statement

The animal study was reviewed and approved by Institutional Animal Care and Use Committee of Jilin University, IACUC, No. 2019JLU23D.

## Author Contributions

YQ and JZ conceived and designed the experiments. MK and XC performed the experiments and analyzed data. YQ and JZ wrote the manuscript. All authors contributed to the article and approved the submitted version.

## Conflict of Interest

The authors declare that the research was conducted in the absence of any commercial or financial relationships that could be construed as a potential conflict of interest.
